# Intervention of Fluency and Anxiety in Mindfulness Training of Shooting

This article has been retracted.

**DOI:** 10.1155/2022/6069561

**Published:** 2022-04-26

**Authors:** Wei Liu

**Affiliations:** School of National Security, People's Public Security University of China, Beijing 100038, China

## Abstract

**Introduction:**

Mindfulness cognitive therapy is based on mindfulness decompression, integrating the elements of cognitive behavioral therapy and related psychological education components, a set of mindfulness group courses designed.

**Objective:**

In order to explore the influence of mindfulness training on fluency and anxiety in shooting sports training.

**Methods:**

There are 22 athletes in a provincial shooting team, 12 in the experimental group and 10 people in the control group, grouped according to the random principle. A single-participant experiment design with multiple baseline levels of ABA was adopted.

**Results:**

The fluency state of the athletes has increased from 28.75 to 30.63; the average value before the intervention increased by 6.5%, PEM = 88%, explaining that the previous intervention has a moderate-intensity effect. The average value of athletes' sports competition anxiety state 205 before intervention was reduced to 171.25, reduced by 16.5%, PEM = 100%, showing that the intervention effect is very effective.

**Conclusions:**

After the shooting athletes received the intervention of the mindfulness cognitive intervention method MBCT, the state of fluency is improved, the level of competition anxiety is reduced, and the experimental intervention basically confirmed the research hypothesis. This study confirms the moderating role of emotion regulation self-efficacy between mindfulness and the fluency of shooters and provides further impetus for the refinement and development of a push-up spiral model that explains mindfulness mechanisms.

## 1. Introduction

Mindfulness-based cognitive therapy (MBCT) is based on mindfulness decompression, integrating the elements of cognitive behavioral therapy and related psychological education components, a set of mindfulness group courses designed. After MBCT was launched more than ten years ago, it has received a lot of clinical and laboratory research support [1]. Mindfulness cognitive therapy is built on two important sources: intensive mindfulness practice derived from eastern traditional wisdom and modern western cognitive behavioral therapy. Although the two belong to two systems, there are common goals: understand people's hearts and reduce or alleviate mental distress. People's susceptibility is an overreaction to low mood; this often manifests itself in two ways: experience avoidance—try to avoid unwanted experiences; rumination of the mind is to use the mind to solve the problem of the mood [2]. Shooting is a static, nonconfrontational project, requiring a high degree of concentration. And the fluency state can get rid of distracting thoughts, a “peak experience” in which full attention is paid. In this state, athletes can devote themselves to the activities they engage in, in order to enter a state of personal stability, both internal and external interfering athletes can be automatically shielded. And it can let athletes in the process of training or competition immerse in the fun of the activity itself and have a sense of control over the action process [3, 4]. Many studies have shown that mindfulness helps promote fluency experience. Mindfulness includes awareness and conscious attention to the experience of the moment, in a way that does not require judgment and acceptance. Survey shows the challenge of a high degree of mindfulness and fluency experience—technical balance, clear goals, clear physical feedback, attention, awareness of action, and disinterestedness; these six dimensions are closely related [5]. These tasks are much simpler for athletes to understand the concepts than they actually do, and mindfulness training can guide them through the mental skills they need to successfully build.

## 2. Method

### 2.1. Research Objects

22 athletes were from a provincial shooting team (9 males and 13 females), 12 people in the experimental group and 10 people in the control group, grouped according to the random principle. Due to the loss of training athletes and the effectiveness of the athlete's questionnaire, the participation attitude issues lead to the loss of subjects; a total of 14 shooters (3 males and 11 females) completed the entire intervention plan. Age range is 15-31, with average age 22. The training period is 2-20, and the average training period is 9. The grouping situation is as follows: 8 people in the experimental group (2 males and 6 females, with an average age of 22.3 ± 5.7 and an average training period of 8.5 ± 5.6) and there were 6 people in the control group (1 male and 5 females, with an average age of 21.3 ± 6.9 and an average training period of 8.7 ± 6.1). There was no difference in the level of athletes between the experimental group and the control group.

### 2.2. Research Tools

Simplified dispositional flow scale (SDFS): there are 9 questions in this short form; each item is used to measure one of the 9 dimensions of fluency, through the fluency experienced by the subjects in a given situation (such as training and competition situations), and use the 5-point scoring method to answer. The internal consistency reliability of the scale is *a* = 0.70, and the test-retest reliability is *r* = 0.70.

### 2.3. Data Collection and Statistics

Respectively, on the first (start of intervention), third, fifth, seventh (end of intervention) [6], and fifteenth weeks (tracking test), use the Chinese Mindfulness Questionnaire (CMSS) for athlete training games, measure the participant's mindfulness level, use repeated measures analysis of variance to test the effect of the intervention, and analyze the changes in the level of mindfulness of shooting athletes.

### 2.4. Mindfulness Training Methods

During the seven weeks of mindfulness training, select the time points of the first, third, fifth, and seventh weeks, respectively; measure the mindfulness level of the shooter, and in the eighth week (that is, the fifteenth week) after the training, a follow-up test will be conducted. The Chinese Mindfulness Questionnaire (CMSS) was used to measure training and competitions for athletes. In the testing process of mindfulness training, according to the principle of voluntariness and balance, divide all athletes who participated effectively into an experimental group of 8 people and 6 people in the control group.

## 3. Results

### 3.1. Analysis of the Effectiveness of Mindfulness Training

The data will be measured in the first, third, fifth, seventh, and fifteenth weeks, stored in the data file with five variables *t*1~*t*5, respectively, and in accordance with the method and procedure of repeated test analysis of variance, the analysis was carried out in the Chinese version of SPSS 18.0.

First, the existence of a correlation between the repeated measurements was determined by the results of the spherical test.

Immediately after the second step, analyze the role of time and grouping factors and the interaction between time and grouping; the calculation results of the variation part in each body show that the time factor is statistically significant (*P* < 0.05), explaining that the measurement index has a tendency to change over time. But the interaction between time and grouping is close to significant (*P* = 0.055), explaining that the role of the time factor varies with different groups. The calculation results of the variation part between the groups are shown (see Table 1); the statistical significance of the grouping effect is not significant (*P* > 0.05), explaining that the grouping factor does not work; the difference of mindfulness intervention between the experimental group and the control group was not obvious.

With the help of the Plots submenu, the repeated measurement indicators of St are all trend graphs, which can intuitively see the change trend of the measurement index over time, as shown in Figure 1. It can be seen from the figure that starting from the third test (that is, the fifth week), compared with the control group, the experimental group has a significant improvement in the level of mindfulness; in the fourth test (that is, the seventh week), the level of mindfulness continued to be high.

In the follow-up test (the fifteenth week), the mindfulness level of the experimental group had a downward trend, while the control group did not change significantly.

### 3.2. The Role of Self-Efficacy in Emotional Regulation between Mindfulness and Fluency

The fluency score of the athletes is shown in Figure 2.

Figure 2 shows the scores of athletes in the trait fluency state. From the preintervention average of 28.75 to 30.63, increased by 6.5%, PEM = 88%, it shows that the previous intervention has a moderate-intensity effect. The score span has increased from 26-30 to 25-33; it shows that the fluency state of the athletes still fluctuates greatly during the 8 weeks of intervention. In particular, in the 4th week of the intervention, the fluency score dropped significantly, because that week the athlete's emotional dissatisfaction affected his mood. In the later follow-up investigation, the average value was 35.34, an increase of 22.9% compared to before the intervention, PEM = 100%; it shows that the intervention effect is significant. The score span has been shortened from 25-33 to 35-36, and the fluency state is more stable than expected. And the scores are higher than the baseline value, indicating that the intervention has a good sustained effect. The scores of athletes in the anxiety state of sports competitions are shown in Figure 3.

The scores of athletes in the anxiety state of sports competitions are shown in Figure 3. From the preintervention average 205 to 171.25, a decrease of 16.5%, PEM = 100%, showing that the intervention effect is very effective. The score span increased from 190-220 to 150-190; it shows that the athlete's anxiety state is relatively unstable during the intervention period; mood swings are greater. As shown in the figure, in the athletes in the first 3 weeks of the intervention, the effect of improving anxiety is not obvious; starting from the 4th week, the anxiety value has been greatly reduced and continues to maintain a stable state. In the follow-up survey, the average was 166.67; it was 18.7% lower than before the intervention, PEM = 100%, and the anxiety value is higher than the baseline value, indicating that the intervention effect is significant. The score span has been shortened from 150-190 to 160-170; it shows that the anxiety level maintains a relatively stable state, and the intervention has a good sustained effect.

## 4. Discussion

The above analysis results show that the level of mindfulness of shooting athletes has increased significantly, that is, the time factor is significant. The interaction between time and grouping is close to significant, indicating that grouping has a certain effect. And to examine the effect of grouping separately, it shows that the effect is not statistically significant [7, 8]. This shows that the whole seven weeks of mindfulness training has its effect, and to examine the effects of grouping factors separately, statistically significant, it may be due to the following reasons. (1) The control group was followed up with relevant questionnaires; athletes with strong learning and comprehension ability can also learn in the questionnaire; the measured level of mindfulness will increase; this is an invisible learning. (2) Due to the characteristics of athlete management, the control group members who get along day and night may inquire about learning related content in the experimental group members; this is a phenomenon similar to “stealing.” (3) Although some mindfulness exercises will be done in the training class, the team members rarely did mindful breathing and body scanning exercises after class, so, at most, it is just a clarification of cognition in class, or the guidance of some adjustment methods is working, and the athletes did not experience the process of actively internalizing mindfulness practice, so as shown in Figure 1, in the follow-up test, the mindfulness level of the experimental group decreased, while that of the control group hardly changed [9]. This time between mindfulness and the fluency of shooting athletes introduce emotion regulation self-efficacy as a regulation variable, and the interaction with mindfulness affects the fluency state [10].

## 5. Conclusion

The author tries to examine shooting athletes through experiments; after receiving the mindfulness cognitive therapy intervention method, the fluency state can be improved, and the level of competition anxiety has been reduced. From the “simplified trait fluency scale” experimental data analysis, PEM effect analysis, and data analysis of social validity evaluation, all provided support for the intervention effect of this study, it shows that the intervention effect is significant and has good sustainability.

## Figures and Tables

**Figure 1:** The trend chart of the mean change of the 5*t* repeated measurement index in each group.

**Figure 2:** Fluency score.

**Figure 3:** Score of anxiety state in sports competition.

**Table 1:** Calculation results of the variation part between groups.

Source	Type IV sum of squares	df	Mean square	FS	Sig.
Intercept	111723.822	1	111723.822	1815.317	0.000
Grouping	18.404	1	18.404	0.217	0.473
Error	727.156	11	60.413		

## Data Availability

The data used to support the findings of this study are available from the corresponding author upon request.
